# Museum Relic Image Detection and Recognition Based on Deep Learning

**DOI:** 10.1155/2022/9670191

**Published:** 2022-01-24

**Authors:** Qi Wang, Ling Li

**Affiliations:** ^1^Taiyuan R & D Center, Beijing Green Rock Technology Development Co., Ltd, Taiyuan 030051, Shanxi, China; ^2^College of Big Data, North University of China, Taiyuan 030051, Shanxi, China

## Abstract

To improve the accuracy of museum cultural relic image recognition, the DenseNet and ResNet are selected as the backbone neural networks for detection and recognition. In view of the small target problem in cultural relics, the feature pyramid is introduced in this paper to improve the DenseNet method. The accuracy of target detection is improved through multiscale feature extraction and fusion. At the same time, aiming the problem of weak robustness and feature extraction of cultural relic images, the attention mechanism is proposed to improve ResNet. Therefore, this network can pay attention to the key of feature areas in the image. Finally, the aforementioned methods are verified by experiments. The results show that compared with the YOLOv3 and other algorithms, the accuracy of the improved ResNet proposed in this experiment is above 90%. Furthermore, the number of missed and erroneous detection is the lowest, which are 171 and 134, respectively. The identified mAP indicator accuracy can reach 86%, which also exceeds SVD-Net and DenseNet. It can be seen that the constructed method can effectively detect and recognize the museum cultural relic images.

## 1. Introduction

With the continuous development of archaeological work, the number of cultural relics is increasing. How to effectively manage a large number of cultural relics has become the focus of current thinking and research. To solve this problem, modern information technology is introduced. With the progress of artificial intelligence and image processing technology, it provides rich reference for the recognition of cultural relic images. For example, LiMiao Deng et al. used SVM to classify agricultural pest images, which is based on the extraction of agricultural images by SIFT. It can be seen that the types of agricultural pests and diseases can be accurately obtained [1]. Cheng Luo et al. applied YESNet to the video advertising images to detect and identify the advertising images, which greatly improved the correlation with advertising database [2]. Elham Mohammed Thabit A and others reviewed the detection and recognition methods of animal images, including the widely used algorithms, such as SVM, BP, CNN, and RNN. It can be seen that a more macro understanding was provided for image detection and recognition [3]. Loris Nanni et al. adopted biological heuristic algorithm to preprocess the image. Then the teaching plan set neural network was introduced to train the image. So the classification of different pest images can be achieved [4]. Shizhao Zhang et al. directly applied YOLOv3 to the detection and recognition of aviation images. The result showed that this method can effectively improve the accuracy and speed of classification [5]. Zhang Jiaming and others combined lightweight network model with RGB image to improve the accuracy of image detection and recognition [6]

It can be concluded from the aforementioned research that the methods of image detection and recognition are mainly to extract image features and then use convolution neural network and other algorithms to classify those features. However, the aforementioned research indicates that to improve the accuracy of classification is the trend of current research. At the same time, organizing the current periodical databases, it is found that there are few studies on the detection and recognition of museum cultural relic images. For example, Li Pengong et al. only used the method of spatial analysis to analyze the similarity of cultural relics [7]. Therefore, based on the aforementioned theoretical knowledge and application practice of image detection and recognition, a method of museum cultural relic detection and recognition based on convolution neural network is proposed, so as to provide more reference for museum cultural relic recognition.

## 2. Multiscale Detection of Cultural Relics Based on Feature Pyramid

### 2.1. Backbone Network Selection

The backbone network is basic, which can realize the effective extraction of depth features and be applied to subsequent learning tasks. Therefore, to design the backbone network reasonably first is necessary. Currently, there are many researches in this field, and some scholars have proposed different network types, including DenseNet and VGG16, which have differences in specific structure and applicability [8,9]. Although ResNet network can obtain more semantic features, it is easy to lose some effective features by adopting additive method in feature fusion, affecting the effect of the application. Although Inception and VGG16 networks can preserve spatial features, there are also deficiencies and hard to be effectively applied to deep semantic feature extraction. In addition to the aforementioned networks, as the application of DenseNet network adopts the splicing method in the process of feature fusion, retaining the features of each layer has certain advantages. Therefore, DenseNet network is adopted in this design, and the specific structure is as follows [10].

### 2.2. The Network Structure Design

It can be seen from the network structure in Figure 1 that multiple down-pooling layers have been passed in the learning process, resulting in low resolution and low size of the feature maps finally obtained. At the same time, neural network can only detect images of the same size. For some special scenes, such as museums and others, due to the multiple types of cultural relics and significant differences in scale, if the traditional neural network is directly used, it is bound to have poor effect. This is mainly because it increases the difficulty of small-scale object detection and reduces the accuracy of detection results by passing the down-pooling layers. In view of the aforementioned problems, some scholars propose a network based on feature pyramid. By taking advantage of middle layer of the backbone network of feature pyramid network and at last the output of the feature maps learning, feature maps with multiple resolutions are fused to improve the accuracy of target detection. In addition, it is also found in practice that adding the FPN network can improve the ability of multiscale target detection. For example, in FPN network structure, up-sampling of low-resolution features is carried out in feature fusion, and then high-resolution features are added to achieve the target of feature fusion. However, there are still defects in this method, mainly reflected in the following three aspects: First of all, dimension reduction is required for multiscale features. In this process, some feature information is lost; Second, not all of the information in the feature pyramid can be used in feature fusion, but only the current and adjacent scale feature information can be used; Third, as there is a significant gap between feature information of different scales, and direct sum cannot maintain a high-expression ability, it is necessary to screen. Combined with the aforementioned analysis, it can be seen that the expected results cannot be achieved by directly applying the feature pyramid network to the detection of cultural relics. Therefore, a new feature fusion method is proposed, and the specific network structure is shown in Figure 2 [11]. The effect of the network structure in Figure 2 is that we can not only learn a lot of information, but also improve the expression ability of feature graph.

In the cultural relic target detection network shown in the figure, each layer represents a scale feature extracted from the DenseNet backbone network. By subsampling the DenseNet backbone network four times, fusing the features, and then training the network, the deep features can be received. In the fusion process, first, the same scale, which is up-sampled from the features of each scale, is carried out through the 1 × 1 convolutional layer for feature mapping, and nonlinear activation function is introduced into ReLU function, so that the network has stronger feature expression ability; second, feature fusion is carried out by splicing channel dimensions; at last, after the fusion is completed, the corresponding feature map is obtained, and the functions are activated during this process by two convolution layers and Sigmoid.

Through the aforementioned fusion, the deficiency of traditional DenseNet network is made up. On one hand, the effective detection of multiscale features is realized, and each scale feature contains both original information and deep information, improving the network feature extraction ability; on the other hand, it improves the feature extraction and utilization ability of pyramid structure and solves the problem of significant scale change in the detection of cultural relics, so as to improve the accuracy of the detection results of cultural relics.

### 2.3. Loss Function Design

The rationality of the design of loss function will directly affect the effect of network learning, especially on the training efficiency and direction. In this study, GioULoss function is adopted, and FocalLoss function is used in bounding box training. Based on this method, the accuracy of target bounding box detection is improved. It is found in the training that although L1Loss and L2Loss functions are mostly used, the former cannot be differentiated at the zero position and cannot be propagated backward, while the latter is susceptible to the influence of outliers, reducing the stability of the training process. To effectively solve the aforementioned problems, some scholars came up with smooth L1Loss function, and the specific formula is as follows [12, 13]:

(1) $$\begin{array}{c} \text{SmoothL}1=\left\{\begin{array}{c} 0.5x^{2},\;\left|x\right|<1,\\ \left|x\right|-0.5,\;\left|x\right|\geq 1. \end{array}\right. \end{array}$$

Through formula (1) of L1, L2 is improved; however, in error calculation, each value of bounding box coordinates is used, and the relationship of coordinates is ignored, so that the accuracy of the prediction bounding box is reduced. Later scholars come up with IoULoss function, which adopts the IoU of bounding box prediction results and real results. The specific formula is as follows [14]:

(2) $$\begin{array}{c} \text{loU Loss}=1-\frac{\left|A\cap B\right|}{\left|A\cup B\right|}. \end{array}$$

In formula (2), *A* and *B*, respectively, represent the predicted value and actual value of the bounding box. In the case that *A* and *B* are basically consistent, it corresponds to a smaller loss function. However, if there is no overlapping area between *A* and *B*, then the quality of training (IoU) will be reduced. Considering the aforementioned problems, GIoULoss function is adopted in this study, and its formula is as follows [15]:

(3) $$\begin{array}{c} \text{GIoU}=\frac{\left|A\cap B\right|}{\left|A\cup B\right|}-\frac{\left|C-\left(A\cap B\right)\right|}{\left|C\right|},\\ \text{GIoU loss}=1-\text{GIoU}. \end{array}$$

In the aforementioned formula, *C* represents the minimum rectangle of the two bounding box. In the training process of this function, the overlap relation and distance relation of *A* and *B* are fully taken into account, and the loss value can also be obtained for nonoverlapping areas, thus realizing the effect of back propagation. The aforementioned relationship can be illustrated in Figure 3 [16].

### 2.4. Background Region Separation

In the process of target detection, in order to achieve high precision, in addition to the prediction of the position of the bounding box, it is also necessary to separate the target from the background area, so as to obtain the accurate information of the target. However, in fact, the background area is obviously larger, while the target area is relatively small, which leads to the misunderstanding that the bounding box belongs to the background area in the prediction process, that is, the problem of sample imbalance exists. In view of the aforementioned problems, FocalLoss function is selected for classification. In fact, the function improves the cross-entropy cost function with weight; that is, a dynamic adjustment mechanism is added, which can adjust the weight in real time in the network, so as to improve the training effect. The specific formula is as follows [17]:

(4) $$\begin{array}{c} \text{Focal Loss}=-\alpha y{\left(1-p\right)}^{\gamma }\log\;p-\left(1-a\right)\left(1-y\right)p^{\gamma }\log\left(1-p\right). \end{array}$$

In the aforementioned formula, the negative sample containing only background represents the prediction result; *y* stands for training tag; *γ* stands for attenuation coefficient, and if the value is large, it means that the loss attenuation rate is small. If the training effect of the sample is better, it corresponds to a smaller attenuation coefficient, that is, the attenuation speed increases. Based on this method, the problem of unbalanced samples is solved effectively. Therefore, the final adopted loss function is as follows [18]:

(5) $$\begin{array}{c} \text{Loss}=\text{GloU Loss}+\text{Focal Loss.} \end{array}$$

## 3. Cultural Relic Recognition Based on Self-Attention Concentration

The attention mechanism can make the neural network of deep learning pay more attention to a certain area of the image or feature for key learning. At the same time, the attentional mechanism can allocate limited computing resources to the image regions or features that need to be learned. This method uses attention mechanism network to extract useful important information and ignores irrelevant information, which reduces the influence of noise and improves the robustness of feature. The cultural relic identification method based on self-attention mechanism will be introduced in detail.

In the deep learning network, when the convolution kernel performs feature extraction on the image, the learning of each pixel in the image is equivalent. The attention mechanism can concentrate the neural network learning in a certain area, which can greatly reduce the learning time of the neural network. In other words, attentional mechanisms focus on key information, filter and ignore irrelevant information, and ultimately improve feature robustness. Therefore, in order to improve the efficiency of deep learning algorithm, attention mechanism is introduced to identify and classify cultural relics.

In general, when using convolutional neural network, the target's apparent features need to be determined first. In this case, the features of the full-connection layer before classification are mainly used, and adjustments need to be made according to specific recognition requirements. Therefore, in terms of extracting epigenetic features, some scholars proposed twin CNN network to find the best method to distinguish different cultural relics. The basic structure of twin CNN network is shown in Figure 4 [19]. Twin CNN network also has some shortcomings, that is, the introduction of noise reduces the ability of feature expression.

Therefore, based on the aforementioned problems, this study uses the twin CNN network as a foundation and is combined the self-attention mechanism, extracting key epigenetic features and improving the accuracy of classification results.

### 3.1. Cultural Relic Feature Extraction Network Based on Self-Attention Mechanism

At present, attention mechanism is generally divided into supervised and unsupervised, and they have some differences in the generation mode of attention graph. The former uses some measures like manual annotation to generate the key mask of the target region and then obtains the corresponding attention graph. In this process, Sigmoid or Softmax layer is commonly used. In essence, this kind of attention mechanism needs to set up new branches of the backbone network and then multiply the resulting weights with the features of the main branch. The mechanism of self-attention is obviously different because in the generation of self-attention graph, feature map transpose multiplication method is used to realize the constraint on the features of backbone network. In addition, self-attention graph can learn the context of the target image, so as to obtain more valuable information.

In this study, attention graph is adopted, and the specific way of application is through the nonlocal self-attention mechanism, to improve attention to key regions. The basic principle of this mechanism is shown in Figure 5 [20]. Combining with the information shown in the figure, it can be seen that a self-attention module is extended in the backbone network, and it can multiply the generated self-attention graph and the branch network feature graph to obtain the predicted results.

The specific calculation process is as follows.

First, feature map mapping is conducted. At this point, 1 × 1 convolution of three unshared weights is used to obtain the feature graph expressed as *F*_Query_, *F*_Key_,  and *F*_value_, and then the self-attention graph is obtained through the first two feature graphs, and the specific formula of attention value is as follows [21–23]:

(6) $$\begin{array}{c} \beta_{i,j}=\frac{\exp\left(S_{ij}\right)}{\sum_{i=1}^{Tf}\exp\left(S_{ij}\right)},\\ S_{ij}=F_{q}{\left(X_{i}\right)}^{T}F_{K}\left(X_{i}\right), \end{array}$$

and then the feature graph *F*_org_^att^ with the mask is further obtained, and now it has to take the product of *β*_*i*,*j*_ and *F*_value_, and the specific formula is as follows [24]:

(7) $$\begin{array}{c} F_{\text{org}}^{\text{att}}=\sum_{i=1}^{Tf}\beta_{i,j}F_{\text{value}}. \end{array}$$

After the aforementioned process is completed, *F*_org_ and *F*_org_^att^ need to be added to obtain the backward-propagating feature graph *F*_*SA*_, and the specific formula is as follows [25]:

(8) $$\begin{array}{c} F_{SA}=\theta F_{\text{org}}^{\text{att}}+F_{\text{org}}. \end{array}$$

In the aforementioned formula, *θ* represents the adjusting parameter.

In feature extraction, ResNet is used. The input in the network is the cultural relic image after clipping. After feature extraction, the optimized feature graph of the self-attention graph is obtained, and then the classification training is carried out. At this time, the deep-seated features need to be obtained through global average pooling. In the classification, the cross-entropy function is chosen. The basic structure of the network is shown below [26]:

### 3.2. Cultural Relics Feature Distance Measurement

In the field of classification, apparent features similarity is widely used. Based on the distance of apparent features, the similarity between two targets can be calculated, and for example, the commonly used Euclidean distance (Euclidean distance) adopts this principle. This method has high integrity of measurement space and is widely used in feature distance measurement. The specific mathematical principles are as follows:

The eigenvectors *A*(*a*_1_, *a*_2_,…, *a*_*n*_) and *B*(*b*_1_, *b*_2_,…, *b*_*n*_) are known, and the Euclidean distance between them is expressed as *d*_euc_(*A*, *B*), and the specific formula is as follows [27]:

(9) $$\begin{array}{c} d_{\text{euc}}\left(A,B\right)=\sqrt{\sum_{i=1}^{n}{\left(a_{i}-b_{i}\right)}^{2}}. \end{array}$$

Through practice, it is found that there is a problem of inconsistent scale in the application of Euclidean distance, and in the process of calculating similarity, Euclidean distance is very easy to be affected by factors, such as feature dimension, so that accurate calculation results cannot be obtained in some scenes. Therefore, Mahalanobis distance *d*_mah_(*A*, *B*) is often used to solve the aforementioned problems; the formula is as follows:

(10) $$\begin{array}{c} d_{\text{mah}}\left(A,B\right)=\sqrt{{\left(A-B\right)}^{T}\sum^{-1}\left(A-B\right)}. \end{array}$$

Under certain conditions, Mahalanobis distance and Euclidean distance are consistent, that is, if the covariance matrix belongs to the unit vector, each dimension in the vector satisfies the independently identical distribution condition, then the conversion between Mahalanobis distance and Euclidean distance can be realized. Although Mahalanobis distance has high accuracy in feature similarity description, the calculation process is too complex and inefficient, which limits its application. In addition to Euclidean distance, cosine distance is also a common method. When calculating similarity, this method actually uses the cosine value of the angle between feature vectors. Therefore, when the dimension is large, the results of feature vector measurement are: 1 and −1, respectively, when the vectors are the same and opposite, respectively, and equal to 0 when the vectors are orthogonal. The formula is as follows:

(11) $$\begin{array}{c} d_{\cos}\left(A,B\right)=1-s_{\cos}\left(A,B\right)\\ =1-\frac{\sum_{i=1}^{n}a_{i}b_{i}}{\sqrt{\sum_{i=1}^{n}a_{i}^{2}}\sqrt{\sum_{i=1}^{n}b_{i}^{2}}}. \end{array}$$

According to the aforementioned formula, the distance is actually in the range of 0 to 1. The similarity between targets can be calculated by cosine distance, so as to describe the difference between different types. In addition to the aforementioned advantages, this method also solves the problem of dimensional inconsistency, so it is widely used in similarity evaluation.

Combined with the aforementioned method, it can be seen that the single measurement method often has shortcomings. Therefore, the weighted sum of cosine distance and Euclidean distance is adopted in this study. The specific steps are: First, the cropped target image is obtained; then, the target features and image features are compared, and the type of cultural relics can be determined according to the set threshold *T*. The specific formula is as follows:

(12) $$\begin{array}{c} d\left(A,B\right)=ad_{\text{euc}}\left(A,B\right)+\beta d_{\cos}\left(A,B\right). \end{array}$$

## 4. Test Verification

### 4.1. Experimental Environment

The experiment will be carried out according to the method of this design. In the experiment, the necessary environment needs to be configured first, which is mainly divided into two parts: hardware and software. The hardware information is shown in Table 1 [27].

The software part mainly involves application software, system software, and deep learning tools, including PyTorch framework, Pycharm tool, Python language, and Ubuntu 16.04.

### 4.2. Cultural Relics Object Detection Experiment Based on Feature Pyramid

#### 4.2.1. Construction of Training Set

Currently, in the process of network, training can use different data sets, and commonly used ones include COCO, and so on. Such data sets provide rich sample information and meet the requirements of many algorithm tests and applications. However, the detection of cultural relics in this study has certain particularity, and the lack of cultural relic targets in these data sets makes it difficult to achieve good results in the training. Therefore, the data set is constructed by us in this study, and the images are adopted from a museum.

The total number of images collected this time is 4000, which is divided into three parts, namely, training set, test set, and verification set, and the ratio of the three is set as 7:2:1. The collected data are marked, and corresponding labels are obtained using VOC format, which is convenient for training and verification. In addition, there are a variety of cultural relic distributions in the image, and the lighting conditions are different, which meets the basic requirements of cultural relics target detection.

The collected images will be saved, and all information is placed in three paths: JPEGImages, ImageSets, and Annotation, and the specific information in each path is different. The annotation information of the image and other basic information are saved in json. In addition, JPEGImages mainly stores all the original images, and ImageSets stores the configuration file of the data set partition, which is in txt format (Figure 6).

The collected image data set has been used in this experiment, and some images are shown in Figure 7 [28]. The collected data set contains abundant images, and the scene and other factors are taken into comprehensive consideration, which meets the basic requirements of the experiment and can detect the effectiveness of the algorithm. The number of images in the test set reaches 1000, and the number of cultural relic targets involved exceeds 3000. Based on the data set, the application effect of the algorithm has been tested and analyzed and then has been evaluated quantitatively through scientific indicators (Figures 8 and 9).

#### 4.2.2. Evaluation Method

The indicators used in this study include accuracy, precision, and recall, which represent average accuracy, recall rate, and accuracy, respectively. The basic definitions of each indicator are as follows:

The precision refers to the proportion of the real cultural relic target bounding box in all detection bounding boxes. The calculation formula is as follows:

(13) $$\begin{array}{c} \text{precision}=\frac{TP}{TP+FP}. \end{array}$$

Recall rate refers to the proportion of accurate bounding boxes in all real bounding boxes. The formula is as follows:

(14) $$\begin{array}{c} \text{recall}=\frac{TP}{TP+FN}. \end{array}$$

The average accuracy can be obtained on the basis of the aforementioned two indicators, and this average accuracy is actually the average composition of precision under multiple recall. Based on these indicators, the performance of the algorithm can be quantitatively analyzed.

In order to verify the application effect of the design algorithm, it is compared with several other detection methods, including YOLOv3, and then, from two perspectives of qualitative and quantitative analysis, the application effect of the design algorithm of cultural relics object detection will be expounded.

#### 4.2.3. Target Detection Results

The application effect of the algorithm is evaluated by quantitative indicators and then it is compared with other types of algorithms, including precision AP and then the number of false detections are compared with the number of missed detections. The final results are shown in Table 2.

According to Table 2, compared with other types of detection methods, the designed method has achieved better results, and the number of false detection and missed detection is also at a low level, 140 and 176, respectively [29]. While AP, precision, and recall reached 90.2%, 95.5%, and 90.3%, respectively, which were significantly higher than the other four methods. Compared with RtinaNet, using the method of this design, the aforementioned three indicators are improved by 8.7%, 5.4%, and 4.7%, respectively, and the number of false and missed detection is significantly reduced by 31 and 81, respectively. Therefore, according to the results of this study, the effectiveness of the design feature fusion method has been verified, which improves the accuracy of cultural relic target detection and helps improve the effect of cultural relic target recognition.

### 4.3. Cultural Relic Recognition Experiment Based on Self-Attention Mechanism

In this experiment, the main purpose is to verify the application effect of cultural relics feature extraction method. Experiments are carried out in combination with the collected samples, and corresponding conclusions are obtained according to the experimental results. In the experiment, the network feature discrimination ability is detected first, and the specific experimental process is shown as follows: At first, the cultural relic target features are extracted based on the data set, then the sample distance is obtained through the method of this design, and the Acc, Recall, F1-Score, and precision in the experiment are obtained based on the threshold. The specific results are shown in Figure 8.

Combined with the Figure 9, it can be seen that the curve range corresponding to this design method is larger, which can prove that the ability of distinguishing cultural relic targets is higher. In addition, according to the score threshold, it can be seen that the method of this design has a high smoothness, that is, it has a high robustness. There is no need to search too much for the optimal threshold when identifying cultural relic targets, so as to ensure high efficiency. In the study, other types of feature extraction methods are used for comparative analysis [30], and the results obtained are shown in Table 3.

It can be seen from Table 3 that the feature-recognition method designed in this study has a significant improvement effect on mAP, which are 82.5, respectively, then it verifies the reliability of the learning network of cultural relics target features, and it is suitable for the application of cultural relics target recognition and classification.

The final recognition effect is shown in Figure 10. According to the information shown in the figure, the recognition accuracy meets the higher requirements, and the influence of external factors, such as illumination is reduced, showing great application potential.

## 5. Conclusion

Through the aforementioned research, it can be seen that the accuracy and recognition effect of cultural relic detection and recognition combined with attention mechanism and pyramid are significantly better than other algorithms, and the effectiveness of the algorithm proposed in this paper proves the feasibility of the algorithm constructed in this study and achieves the expected design goal. However, the aforementioned is only a method of museum cultural relic image recognition, and in addition to pyramid convolution network, it also includes other neural networks. Therefore, this study needs further experiments.

## Figures and Tables

**Figure 1:** The network structure.

**Figure 2:** The neural network structure constructed in this study.

**Figure 3:** Relationship between bounding boxes in GIoU.

**Figure 4:** Twin network structure.

**Figure 5:** Self-attention network structure.

**Figure 6:** Feature extraction based on self-attention network.

**Figure 7:** The sample of cultural relic data set.

**Figure 8:** The score threshold curve of the network.

**Figure 9:** PR curve.

**Figure 10:** The final recognition effect.

**Table 1:** Test environment construction.

Hardware type	Parameter configuration	Software environment	Name
Processor	Intel(R)Core(TM)i7-6700	OS	Ubuntu 16.04
Memory	16 GB	Application software	Pycharm
Graphics card	NVDIAGeForceGTX1070	Computer language	*Python*
Memory capacity	8 GB	Deep learning framework	PyTorch
Memory interface	256 bit		

**Table 2:** Comparison of cultural relics test results.

Method	ACC	Recall	Precision	Number of missed inspections	Number of false detections
MaskR-CNN	69.7	78.4	76.9	327	259
SSD	66.2	79.5	75.8	251	186
YOLOv3	68.7	75.7	75.8	242	212
RetinaNet	81.5	85.6	90.1	257	171
This point	90.2	90.3	95.5	176	140

**Table 3:** The effect of network recognition.

Method	mAP
SVD-net	61.8
DenseNet121	74.7
PCB	78.1
This point	82.5

## Data Availability

The experimental data used to support the findings are available from the corresponding author upon request.
